This article has been retracted.

# Qingyihuaji Formula Inhibits Pancreatic Cancer and Prolongs Survival by Downregulating Hes-1 and Hey-1

**DOI:** 10.1155/2015/145016

**Published:** 2015-12-13

**Authors:** Yanli Xu, Shan Xu, Yueqin Cai, Luming Liu

**Affiliations:** ^1^Department of Integrative Oncology, Fudan University Shanghai Cancer Center, Shanghai 200032, China; ^2^Department of Oncology, Shanghai Medical College, Fudan University, Shanghai 200032, China; ^3^College of Basic Medical Science, Zhejiang Chinese Medical University, Hangzhou 310053, China; ^4^Laboratory Animal Research Center, Zhejiang Chinese Medical University, Hangzhou 310053, China

## Abstract

The dire prognosis of pancreatic cancer has not markedly improved during past decades. The present study was carried out to explore the effect of Qingyihuaji formula (QYHJ) on inhibiting pancreatic cancer and prolonging survival in related Notch signaling pathway. Proliferation of pancreatic cancer cells (SW1990 and PANC-1) was detected by MTT assay at 24, 48, and 72 h with exposure to various concentrations (0.08–50 mg/mL) of QYHJ water extract. Pancreatic tumor models of nude mice were divided into three groups randomly (control, QYHJ, and gemcitabine). mRNA and protein expression of Notch target genes (Hes-1, Hey-1, Hey-2, and Hey-L) in dissected tumor tissue were detected. Results showed that proliferation of SW1990 cells and PANC-1 cells was inhibited by QYHJ water extract in a dose-dependent and time-dependent manner. QYHJ effectively inhibited tumor growth and prolonged survival time in nude mice. Expression of both Hes-1 and Hey-1 was decreased significantly in QYHJ group, suggesting that Hes-1 and Hey-1 in Notch signaling pathway might be potential targets for QYHJ treatment. This research could help explain the clinical effectiveness of QYHJ and may provide advanced pancreatic cancer patients with a new therapeutic option.

## 1. Introduction

Pancreatic cancer remains one of the most common causes for cancer related death all over the world. The prognosis of pancreatic cancer is very poor, and its 5-year survival rate is only 6% [1]. To date, complete surgical resection is still the main therapeutic option, but unfortunately, the majority of patients are diagnosed at a locally advanced or distant metastatic stage, thus precluding surgical cure [2]. Currently available treatment options for advanced pancreatic cancer, such as gemcitabine, always have strong side effects but limited impact on patient survival. Therefore, more effective agents are needed urgently to control this deadly disease.

Qingyihuaji formula (QYHJ), composed of traditional Chinese herbs, has been applied to human pancreatic cancer treatment for many years. Our clinical study indicates that the treatment with QYHJ combined with western medicine has prolonged survival time of advanced pancreatic cancer patients [3–7]. However, its underlying mechanism remains to be elucidated.

It is well reported that loss of normal regulation of cell growth is the main cause of tumorigenesis, development, and metastasis. Notch signaling pathway does play an important role in regulating cell fate decision, cell differentiation, proliferation, and apoptosis [8, 9]. Hes genes and Hey genes are recognized as Notch downstream target genes. In mammals, Hes-1 is the most extensive expressed one of Hes family, and Hey family includes Hey-1, Hey-2, and Hey-L [10–12]. Activation of Notch signaling pathway has been described in several human malignancies, including pancreatic cancer. In normal pancreas, little-to-no expression of Notch signals was detected, while overexpression of Notch related molecules was found in pancreatic cancer [13–16]. Hes and Hey, as important target genes of Notch signaling pathway, could reflect expression level of Notch signals.

Thus, the aim of the study is to investigate both* in vivo* and* in vitro* effects of QYHJ on inhibiting pancreatic cancer and prolonging survival via Notch signaling pathway.

## 2. Materials and Methods

### 2.1. Cell Lines

Human pancreatic cancer cell lines SW1990 and PANC-1 were purchased from American Type Culture Collection (ATCC). The cells were cultured in a humidified 5% CO_2_ atmosphere at 37°C.

### 2.2. Reagents

QYHJ is composed of banzhilian (*Scutellaria barbata*) 30 g, baihuasheshecao (*Hedyotis diffusa*) 15 g, sheliugu (*Amorphophallus rivieri* Durieu) 15 g, jiaogulan (five-leaf* Gynostemma* herb) 30 g, and baidoukou (*Amomum cardamomum*) 3 g. All herbs were purchased from Tianjiang Pharmaceutical Co. (Jiangyin, China). The fingerprint chromatograms of QYHJ for quality control were shown in our previous paper [17]. The daily dosage of QYHJ for nude mice was 36 g/kg according to previous reports [18–21]. Herbs were soaked in distilled water for 30 minutes, boiled in 10 volumes of water for 1 h, and then extracted twice. The final concentration of QYHJ for nude mice was 3.6 g/mL (equivalent to dry weight of raw materials). The final concentration of QYHJ water extract for* in vitro* experiments was 0.31 g/mL (equivalent to dry weight of raw materials), provided by the College of Pharmaceutical Science, Zhejiang Chinese Medical University (Hangzhou, China). Gemcitabine (Eli Lilly) was dissolved in sterile PBS. Antibody against Hes-1 and antibody against Hey-1 were purchased from Abcam.

### 2.3. 3-(4,5-Dimethylthiazol-2-yl)-2,5-diphenyltetrazolium Bromide (MTT) Assay

Inhibition of cell proliferation by QYHJ water extract was measured by MTT assay. SW1990 cells (5 × 10^4^ cells/mL) and PANC-1 cells (5 × 10^4^ cells/mL) were seeded in 96-well plates (100 *μ*L/well) and were incubated at 37°C for 24 h, respectively. Cells were then treated with QYHJ water extract (0.08, 0.4, 2, 10, and 50 mg/mL) for 24, 48, and 72 h. After incubation, 20 *μ*L MTT (5 mg/mL) was added to each well, and plates were kept at 37°C for 4 h in the dark. The formazan was resolved by dimethyl sulfoxide (DMSO), and optical density (OD) was measured at 490 nm by Microplate Reader (BIO-RAD). Cell proliferation inhibition rate was calculated using the following formula:

(1) cell  proliferation  inhibition  rate%=mean  OD  of  control  cells−mean  OD  of  treated  cellsmean  OD  of  control  cells×100%.

### 2.4. Animal Model and Treatment Groups

Male BALB/c-nu/nu mice, five weeks old, weighing 16 g–20 g, were purchased from the Laboratory Animal Research Center, Zhejiang Chinese Medical University. Mice were acclimated for 7 days and were raised in specific pathogen-free (SPF) conditions in separate cages. Local guidelines for the care and use of laboratory animals of Zhejiang Chinese Medical University were followed to carry out experiments in this study.

#### 2.4.1. Pancreatic Orthotopic Transplantation Tumor Model

SW1990 cells (1 × 10^7^ cells in 0.2 mL) were subcutaneously injected into the nape of five nude mice. After growing to a volume of 1 cm^3^, tumor tissues were resected and then cut into small pieces of 1 mm^3^. 24 mice were anesthetized by isoflurane inhalation, and an incision was made in the upper left abdomen of each mouse. The pancreas was exposed, and the small tumor pieces were implanted into the tail of pancreas. The pancreas was then returned to the abdomen, and the peritoneum and skin were closed with a continuous suture. Mice were observed for 24 h after surgery. After 1 week of implantation, mice were divided into three groups randomly (*n* = 8 in each group), using the table of random number: (A) control (treated with water, 10 mL/kg); (B) QYHJ 36 g/kg, once per day p.o.; (C) gemcitabine 25 mg/kg [22, 23], twice per week by i.p. injection. Treatment was continued until mice died.

#### 2.4.2. Subcutaneous Transplanted Pancreatic Tumor Model

SW1990 cells (5 × 10^6^ cells in 0.2 mL) were subcutaneously injected into the nape of each nude mouse. After 24 h of cell inoculation, mice were divided into three groups randomly (*n* = 8 in each group), using the table of random number: (A) control (treated with water, 10 mL/kg); (B) QYHJ 36 g/kg, once per day p.o.; (C) gemcitabine 25 mg/kg, twice per week by i.p. injection. Treatment was continued for 21 days.

### 2.5. Overall Survival Time (Orthotopic Model)

Overall survival (OS) time was recorded from the date of treatment to the date of death.

### 2.6. Assessment of Tumorigenicity* In Vivo* (Subcutaneous Model)

Tumor size was evaluated every 3 days. Tumor volume was measured by the following formula:

(2) $$\begin{array}{c} \text{tumor volume}=\frac{\left(\text{length}\times {\text{width}}^{2}\right)}{2}. \end{array}$$

After 21 days of treatment, mice were sacrificed, and tumors were weighed. Parts of tumor tissues were fixed in 10% neutral buffered formalin and then embedded in paraffin. Tumor growth inhibition rate was calculated by the following formula:

(3) tumor  growth  inhibition  rate%=mean  tumor  weight  of  control  mice−mean  tumor  weight  of  treated  micemean  tumor  weight  of  control  mice×100%.

### 2.7. RNA Extraction and Real-Time Quantitative Reverse Transcription-Polymerase Chain Reaction (RT-PCR)

Total RNA was extracted from equal amounts of all tumor tissue samples using TRIzol Reagent (TAKARA). Aliquots of total RNA (2 *μ*g) were used for RT-PCR according to the manufacturer's protocol (TAKARA). Real-time quantitative RT-PCR analyses were performed in an iCycler iQ system (BIO-RAD), using HotMaster Taq DNA Polymerase (TAKARA) and SYBR Green I (BIO-RAD). The target genes included Hes-1, Hey-1, Hey-2, and Hey-L. GAPDH was included as the internal control. Specific primer sequences were designed (Table 1).

### 2.8. Western Blot Analysis

A 100 mg pancreatic tumor tissue sample from each group was lysed in ice-cold RIPA lysis buffer. Insoluble debris was removed by centrifugation at 10000 rpm for 5 minutes. Aliquots of supernatant protein (200 *μ*g) were separated by 8% sodium dodecyl sulfate-polyacrylamide gel electrophoresis (SDS-PAGE) and then transferred to a nitrocellulose membrane for western blot. Quantification of blot was performed by LI-COR Image Studio Software.

### 2.9. Immunohistochemical Analysis

Paraffin-embedded sections (4 *μ*m) were stained with primary antibodies for Hes-1 (1 : 200) or Hey-1 (1 : 150) and then stained with HRP conjugated secondary antibodies. Sections were developed in diaminobenzidine and counterstained with hematoxylin. Images were taken, and five fields (400x) selected randomly from each section were examined. For the data quantification, integrated optical density (IOD) of positive expression was measured by Image Pro Plus 6.0 software.

### 2.10. Statistical Analysis

Kaplan-Meier analysis was used to evaluate OS, and log-rank test was used to compare OS between groups. Other data were shown as mean ± SD and analyzed by one-way analysis of variance (ANOVA) plus least-significant difference (LSD) test with SPSS 16.0. *P* < 0.05 was considered to be statistically significant.

## 3. Results

### 3.1. MTT Assay

Cell viability was measured at concentrations of QYHJ water extract varying from 0.08 to 50 mg/mL after 24, 48, and 72 h. As shown in Figure 1, both SW1990 and PANC-1 cell growth were inhibited by QYHJ water extract in a dose-dependent and time-dependent manner. At the higher concentration of 50 mg/mL, QYHJ water extract induced significant 89.23% inhibition on SW1990 cells and 78.14% inhibition on PANC-1 cells after 72 h of exposure, respectively. The results indicated that QYHJ water extract has strong antiproliferation activity on both SW1990 cells and PANC-1 cells.

### 3.2. Survival Analysis

Survival time was observed in different treatment groups of pancreatic orthotopic transplantation tumor model. The Kaplan-Meier curves in Figure 2 demonstrated the differences in survival between groups. This showed a significant trend towards improved survival in QYHJ group compared to either control group or gemcitabine group, with median survival time of 38.0, 32.0, and 21.0 days, respectively (*P* < 0.01 compared to control group and *P* < 0.01 compared to gemcitabine group). The survival time of gemcitabine group seemed shorter, although there was no statistical difference compared with control group (*P* > 0.05).

### 3.3. Tumor Growth Inhibition

We evaluated therapeutic effects of QYHJ and gemcitabine on tumor development in subcutaneous transplanted pancreatic tumor model. The results showed a drastic increase of tumor volume in control group compared with other groups (Figure 3). The mean tumor weight of control mice was 0.547 ± 0.174 g, while those of mice treated by QYHJ and gemcitabine were 0.316 ± 0.080 g and 0.262 ± 0.146 g, significantly less than control group (*P* < 0.05) (Figure 3). We noticed that QYHJ effectively inhibited tumor growth within 42.23% tumor inhibition rate (*P* < 0.05), gemcitabine had 52.10% tumor inhibition rate (*P* < 0.05), and no big difference was observed between the two treatment groups (*P* > 0.05).

### 3.4. Gene Expression of Notch Target Genes in Tumor Samples

To investigate whether QYHJ treatment regulated the Notch signaling, we detected mRNA expression of Notch target genes. The results demonstrated that when compared to control, expression of Hes-1 gene and Hey-1 gene was significantly decreased by QYHJ (*P* < 0.01), while gemcitabine had no significant effect (*P* > 0.05). Hey-2 and Hey-L mRNA expression were also examined; however, there were no distinct changes in both QYHJ group and gemcitabine group compared to control group (*P* > 0.05) (Figure 4).

### 3.5. Protein Expression of Hes-1 and Hey-1 in Tumor Samples

Western blot analysis was used to further detect protein expression of Hes-1 and Hey-1. The data in Figure 5 suggested that protein expression of Hes-1 was reduced obviously in QYHJ group compared with control group (*P* < 0.01). Besides, QYHJ treatment was more effective in decreasing protein expression of Hey-1 (*P* < 0.001). However, gemcitabine treatment had no significant influence on protein expression of both Hes-1 and Hey-1 (*P* > 0.05). These results revealed the same tend as real-time quantitative RT-PCR analysis.

### 3.6. Immunostaining Expression of Hes-1 and Hey-1 in Tumor Samples

To explore whether expression of Hes-1 and Hey-1 in tissue level was consistent with those in mRNA level and protein level, we performed immunohistochemistry analysis (Figure 6). The data of IOD indicated that pancreatic tumor tissue in QYHJ treatment group had less immunohistochemical staining of Hes-1 expression and Hey-1 expression as compared to control group (*P* < 0.001), while no statistical difference was found in gemcitabine treatment group (*P* > 0.05). The results further confirmed that expression of both Hes-1 and Hey-1 could be downregulated by QYHJ.

## 4. Discussion

As a result of the poor prognosis, there is a crucial need to improve pancreatic cancer patient survival, although research has shown only limited benefit with current therapeutic options. For over a decade, gemcitabine had been in the first line for treatment of advanced pancreatic cancer patients, while the median survival time was unsatisfactory, approximating 6 months [24, 25].

In China, traditional Chinese medicine has had an advantage in cancer treatment for thousands of years. During the past years, QYHJ has shown promising results in treatment for pancreatic cancer patients. In QYHJ treatment group, the survival rate of 1, 3, and 5 years was 25.0%, 14.1%, and 8.4%, and the median survival time was 7.6 months, obviously longer than that of control group [4]. QYHJ could benefit advanced pancreatic cancer patients by stabilizing tumors and prolonging life expectancy, with fewer side effects than those of chemotherapy or radiotherapy [3, 5]. Another retrospective study also showed that, from January 2002 to December 2007, patients who took QYHJ based integrative treatment have much longer survival, 20 cases survive more than 3 years, of which 13 cases survive more than 5 years, and the longest survival time is 169 months [6]. These studies indicated that QYHJ might be a novel therapeutic option for pancreatic cancer treatment. Therefore, it is valuable to explore its antitumor mechanism.

In this study, we confirmed that QYHJ had obvious advantages in prolonging survival time, which is consistent with our clinical studies. Our results also showed that QYHJ significantly inhibited pancreatic cancer cell proliferation in both a dose-dependent and time-dependent manner* in vitro* and effectively inhibited tumor growth* in vivo*. To further explore the antitumor mechanism of QYHJ, we focused on Notch signaling pathway, which is related to tumor initiation and tumor development in pancreatic cancer.

Multiple factors are involved in regulating Notch signaling. Ligand-binding initiates cleavage of Notch receptors to release Notch intracellular domain (NICD). The NICD translocates to the nucleus and promotes transcription of main Notch target genes including Hes and Hey. Thus, Hes/Hey directly influences cell fate determination as a crucial Notch effector [12].

In previous studies, Notch signaling components and target genes were overexpressed significantly in pancreatic cancer cells [14, 15], and downregulation of Notch genes results in inhibiting cell growth and inducing apoptosis [26, 27]. Moreover, Notch target genes like Hes-1 and Hey-1 were confirmed as prognostic biomarkers in pancreatic cancer; high expression of these genes was associated with shorter overall survival time and progression-free survival time [28, 29]. These findings demonstrate that Notch could be an effective target for pancreatic cancer treatment. In this experiment, we investigated expression of Notch target genes to explore the impact of QYHJ on Notch signaling pathway. We found that QYHJ downregulated Hes-1 expression and Hey-1 expression in both mRNA level and protein level, which was more effective than gemcitabine treatment, indicating that QYHJ may inhibit pancreatic cancer through targeting Hes-1 and Hey-1.

Emerging data have suggested that only a few cells in the malignant tumor, termed cancer stem cells (CSCs), are the main cause of tumor initiation and invasion. The existence of CSCs helps better explain clinical observations that tumor regression may have nothing to do with the survival of patients, because tumor recurrence and metastasis are mainly due to the survival of CSCs [30, 31]. Thus, CSCs play a vital role in predicting prognosis of cancer patients. High levels of CSCs detected in patients lead to poor prognosis [32, 33], and targeting CSCs results in prolonged survival [34, 35].

The strong evidence supporting abnormal Notch signals correlate with the maintenance of CSCs makes Notch be considered as a promising therapeutic target [36, 37]. It was reported that pancreatic CSCs contained increased expression of Notch molecules than nonpancreatic CSCs, and downregulating Notch signaling pathway contributed to a decreased invasive behavior of pancreatic CSCs [38, 39]. Therefore, Notch-targeted therapy might be helpful for eradication of CSCs, which will definitely improve the survival of pancreatic cancer patients. In the current study, QYHJ could prolong the survival time and decrease expression of Notch-targeted genes Hes-1 and Hey-1, indicating that downregulating main target genes in Notch signaling pathway might be its potential mechanism for improvement of survival in pancreatic cancer. However, this work was preliminary; further research will be done in the future.

In conclusion, QYHJ exhibited its significant effect on survival improvement and antitumor activity probably by downregulating related Notch signaling pathway. It is considered that Hes-1 and Hey-1 might be potential targets. This research could help explain the effectiveness of QYHJ and may provide advanced pancreatic cancer patients with a new therapeutic option.

## Figures and Tables

**Figure 1:** Effect of QYHJ on pancreatic cancer cell proliferation. (a) SW1990 cells. (b) PANC-1 cells. QYHJ: Qingyihuaji formula.

**Figure 2:** Effect of QYHJ on survival time of pancreatic tumor nude mice. QYHJ: Qingyihuaji formula; Gem.: gemcitabine.

**Figure 3:** Effect of QYHJ on pancreatic tumor growth (subcutaneous transplanted tumor model). (a) Time-dependent inhibition of pancreatic tumor growth. (b) Mean tumor weight. QYHJ: Qingyihuaji formula; Gem.: gemcitabine. ^*∗*^ *P* < 0.05, compared with control group.

**Figure 4:** Real-time quantitative RT-PCR analyses. (a) Relative mRNA expression of Hes-1. (b) Relative mRNA expression of Hey-1. (c) Relative mRNA expression of Hey-2. (d) Relative mRNA expression of Hey-L. QYHJ: Qingyihuaji formula; Gem.: gemcitabine. ^*∗*^ *P* < 0.01, compared with control group.

**Figure 5:** Western blot analyses on expression of Hes-1 and Hey-1. (a) Protein bands. (b) Relative protein expression of Hes-1. (c) Relative protein expression of Hey-1. QYHJ: Qingyihuaji formula; Gem.: gemcitabine. ^*∗*^ *P* < 0.01, ^*∗∗*^ *P* < 0.001, compared with control group.

**Figure 6:** Effect of QYHJ on expression of Hes-1 and Hey-1 in pancreatic tumor tissues. (a) Immunohistochemical staining for Hes-1 expression in pancreatic tumor tissues (original magnification: ×400). (b) Immunohistochemical staining for Hey-1 expression in pancreatic tumor tissues (original magnification: ×400). (c) Integrated optical density of positive expression about Hes-1. (d) Integrated optical density of positive expression about Hey-1. QYHJ: Qingyihuaji formula; Gem.: gemcitabine. ^*∗*^ *P* < 0.001, compared with control group.

**Table 1:** mRNA specific primer sequences and annealing temperatures.

Gene name	Primer sequences	Annealing temperature
Hes-1 F	5′-TCAACACGACACCGGACAAAC-3′	60°C
Hes-1 R	5′-ATGCCGGGAGCTATCTTTCTT-3′	

Hey-1 F	5′-CCGACGAGACCGAATCAATAAC-3′	60°C
Hey-1 R	5′-TCAGGTGATCCACAGTCATCTG-3′	

Hey-2 F	5′-CGCCCTTGTGAGGAAACGA-3′	60°C
Hey-2 R	5′-CCCAGGGTAATTGTTCTCGCT-3′	

Hey-L F	5′-AAGCGCAGAGGGATCATAGAG-3′	60°C
Hey-L R	5′-GACCAATCGTCGCAATTCAGA-3′	

GAPDH F	5′-TGTGTCCGTCGTGGATCTGA-3′	60°C
GAPDH R	5′-TTGCTGTTGAAGTCGCAGGAG-3′	
